# Acetonic and Methanolic Extracts of *Heterotheca inuloides*, and Quercetin, Decrease CCl_**4**_-Oxidative Stress in Several Rat Tissues

**DOI:** 10.1155/2013/659165

**Published:** 2013-01-10

**Authors:** Elvia Coballase-Urrutia, José Pedraza-Chaverri, Noemí Cárdenas-Rodríguez, Bernardino Huerta-Gertrudis, Mercedes Edna García-Cruz, Hortencia Montesinos-Correa, Dolores Javier Sánchez-González, Rafael Camacho-Carranza, Jesús Javier Espinosa-Aguirre

**Affiliations:** ^1^Laboratorio de Neuroquímica, Instituto Nacional de Pediatría, Insurgentes Sur 3700-C, 04530 México, DF, Mexico; ^2^Departamento de Biología, Facultad de Química, Universidad Nacional Autónoma de México, Edificio F, Segundo Piso, Laboratorio 209, 04510 México, DF, Mexico; ^3^Servicio de Endocrinología, Instituto Nacional de Pediatría, Insurgentes Sur 3700-C, 04530 México, DF, Mexico; ^4^Departamento de Biología Celular, Escuela Médico Militar, Universidad del Ejército y Fuerza Aérea, 11200 México, DF, Mexico; ^5^Departamento de Medicina Genómica y Toxicología Ambiental, Instituto de Investigaciones Biomédicas, Universidad Nacional Autónoma de México 04510 México, DF, Mexico

## Abstract

The present study was designed to test the hypothesis that the acetonic and methanolic extracts of *H. inuloides* prevent carbon tetrachloride-(CCl_4_) induced oxidative stress in vital tissues. Pretreatment with both *H. inuloides* extracts or quercetin attenuated the increase in serum activity of alkaline phosphatase (ALP), total bilirubin (BB), creatinine (CRE), and creatine kinase (CK), and impeded the decrease of *γ*-globulin (*γ*-GLOB) and albumin (ALB) observed in CCl_4_-induced tissue injury. The protective effect was confirmed by histological analysis with hematoxylin-eosin and periodic acid/Schiff's reagent. Level of lipid peroxidation was higher in the organs of rats exposed to CCl_4_ than in those of the animals treated with *Heterohteca* extracts or quercetin, and these showed levels similar to the untreated group. Pretreatment of animals with either of the extracts or quercetin also prevented the increase of 4-hydroxynonenal and 3-nitrotyrosine. Pretreatment with the plant extracts or quercetin attenuated CCl_4_ toxic effects on the activity of several antioxidant enzymes. The present results strongly suggest that the chemopreventive effect of the extracts used and quercetin, against CCl_4_ toxicity, is associated with their antioxidant properties and corroborated previous results obtained in liver tissue.

## 1. Introduction

Oxidative stress describes the level of oxidative damage in a cell, tissue, or organ, caused by reactive oxygen species (ROS) [1]. Various environmental factors such as exposure to environmental pollutants, drugs, UV radiation, and normal cellular activities cause production of ROS such as superoxide radical, hydrogen peroxide, and hydroxyl radical [1, 2]. Under normal circumstances, the generated ROS are detoxified by the antioxidant defenses leading to equilibrium between these two processes. However, owing to ROS overproduction and/or inadequate antioxidant defenses, this equilibrium is hampered favoring a surge of ROS that culminates in oxidative stress. The ROS readily attack and induce oxidative damage to several biomolecules including proteins, lipids, lipoproteins, and DNA [1–3], contributing to the development of various human diseases [2, 3]. Nonenzymatic antioxidants (e.g., glutathione, uric acid, bilirrubin, ascorbic acid, and *α*-tocopherol) help to prevent the damage caused by ROS; additionally, living organisms have developed an enzymatic antioxidant defense system that includes the presence of superoxide dismutase (SOD), catalase (CAT), and glutathione peroxidase (GPx) [2]. It has been reported that good health can be maintained from the consumption of plants with high antioxidant activities [4, 5]. There is some evidence that bioactive compounds and microelements from different functional foods, herbs, and nutraceuticals can ameliorate or even prevent diseases [4–6]. Different reports have established that the industrial solvent, carbon tetrachloride (CCl_4_), is a potent environmental hepatotoxin [7]. The products of CCl_4_ metabolism by CYP2E1 include the highly reactive species trichloromethyl and trichloromethyl peroxy radicals that may produce damage by covalently binding to cellular macromolecules to form nucleic acid, protein, and lipid adducts [7, 8]. Under oxygen rich conditions, the trichloromethyl radical is converted to the more reactive trichloromethyl peroxy radical that can attack polyenoic (polyunsaturated) fatty acids in the cellular membrane initiating subsequent autocatalytic lipid peroxidation related to the disruption of cellular membranes [7]. A number of recent reports clearly demonstrated that the hydrophobic nature of CCl_4_ allows it to permeate cell membranes, and it is distributed and accumulated in different organs, causing disorders in kidneys, lungs, testis, and brain as well as in blood by generating free radicals [7–10]. Due to its well-known toxicity and mechanism of action, we decided to use CCl_4_ as a model environmental toxic substance to test the capacity of *Heterotheca inuloides* extracts to counteract with its free-radical dependent toxicity [11]. Administration of antioxidants from natural sources could protect against free radicals and ROS adverse effects and thereby retard the progress of many diseases [12–14].

In Mexico, more than 90% of the general population use medicinal plants in common practice for the empirical treatment of several diseases [15]. However, most physicians disagree with the use of plant products due to the lack of toxicological and pharmacological studies. In urban areas, prescriptions for medicinal plants are done by vendors of herbal products, whereas in rural areas the populations refer to the local healers, “chamanes,” to receive treatment. 

*Heterotheca inuloides *(Asteraceae) grows abundantly in the cooler and temperate regions of México [11]. The dried flowers of *H. inuloides* known as “arnica” have long been used as a folk medicine for the topical treatment of contusions, bruises, and postoperative thrombophlebitis [16]. More frequently, this plant has been used externally for the treatment of skin wounds and injuries [16, 17]. Furthermore, different metabolites of *H. inuloides* have been recognized as antioxidant [18–20], for its inhibitory activity against lipid peroxidation and oxidative hemolysis [21], anti-inflammatory, analgesic, and cytotoxic effects against several solid tumor cell lines [19, 22] and its antimicrobial activity [23]. In previous *in vivo *experiments we observed that the acetonic and methanolic extracts of *H. inuloides,* and quercetin, displayed hepatoprotective effects against CCl_4_ toxicity in rats [11]. In the present study we show the potential protective effect of acetonic and methanolic extracts and quercetin, the major constituent of *H. inuloides,* in inhibiting CCl_4_-induced damage in different rat organs other than liver. 

## 2. Materials and Methods

### 2.1. Chemicals

Xanthine, nitroblue tetrazolium (NBT), 3,3-diaminobenzidine, bovine serum albumin, xanthine oxidase, nicotinamide adenine dinucleotide phosphate (NADPH), oxidized glutathione (GSSG), reduced glutathione (GSH), trimethoxypropane, 5,5-dimethyl-1-pyrroline-N-oxide (DMPO), hypoxanthine, glutathione reductase (GR), and 2,4-dinitrophenylhydrazine, 1-chloro-2,4-dinitrobenzene (CDNB) were purchased from Sigma-Aldrich (St. Louis, MO, USA). Ethylenediaminetetraacetic acid disodium salt (EDTA), ammonium sulfate, and copper chloride were purchased from JT Baker (México City, Mexico). H_2_O_2_, formaldehyde and sodium carbonate were purchased from Mallinckrodt (Paris, KY, USA). Sodium azide was purchased from Merck (México City, Mexico). Rabbit anti-3-NT polyclonal antibodies were purchased from Upstate (Lake Placid, NY, USA). Mouse anti-4-HNE monoclonal antibodies were purchased from Oxis International, Inc. (Portland, OR, USA). Anti-rabbit IgG horseradish peroxidase antibody and anti-mouse IgG horseradish peroxidase antibody were purchased from Amersham Life Sciences (Buckinghamshire, England). Donkey anti-goat IgG horseradish peroxidase antibodies were purchased from Santa Cruz Biotechnology, Inc. (Santa Cruz, CA, USA). All other chemicals were reagent grade and commercially available.

### 2.2. Plant Material and Extraction

Flowers from aerial parts of* Heterotheca inuloides *were collected in Zacapoaxtla, Puebla, Mexico. The plant material was authenticated by Biol. Myrna Mendoza at the Department of Medicinal Plants of Jardín Botánico (Instituto de Biología, UNAM) and a voucher specimen (Myrna Mendoza C 15,375) is kept in the Ethnobotanical collection of the National Herbarium at Instituto Mexicano del Seguro Social (IMSS) (México City). The quercetin isolated from the methanolic extract of *H. inuloides *was provided by Dr. Guillermo Delgado (Instituto de Química, Universidad Nacional Autónoma de México, Mexico). Dried and powdered plant material (2.0 kg) was extracted with acetone at room temperature (3 times/24 h) followed by methanol extraction (3 times/24 h), to afford, after solvent evaporation, 12 and 15 g of residue, respectively [22]. Acetone extract residue was dissolved in olive oil and methanolic extract residue and quercetin in phosphate buffer pH 7.4 prior to oral administration to rats. 

### 2.3. Total Polyphenols and Flavonoid Determinations

#### 2.3.1. Determination of Total Polyphenols

 Total polyphenols were determined in the acetonic and methanolic extracts by the Folin-Ciocalteu method [24]. 0.1 mL of each extract solution containing 100 mg plant extract was mixed with100 *μ*L of Folin-Ciolcateu reagent. The mixture was incubated for 1 min at room temperature, and 300 *μ*L of sodium carbonate (200 g/L) was added. The mixture was incubated for 15 min at 50°C and cooled in a water ice bath. Finally, the absorbance at 765 nm was scored in a spectrophotometer (Model Year 2000 compliant. He*λ*ios *α*, Cambridge, UK). Total polyphenols were expressed as mg of catechin equivalents/g of extract after extrapolating in a calibration curve obtained following the same procedure described above and using *α* (+)catechin and quercetin as standard.

#### 2.3.2. Analysis of Flavonoid Content

Total quercetin in acetonic and methanolic extract was determined with aluminium chloride (AlCl_3_) [25]. The plant extract (0.1 mL) was added to 0.3 mL distilled water followed by NaNO_2_ (0.03 mL, 5%). After 5 min at 25°C AlCl_3_ (0.03 mL, 10%) was added. The mixture was incubated for 5 min at room temperature and 0.2 mL 1 mM NaOH. Absorbtion at 510 nm was scored in a spectrophotometer (Model Year 2000 compliant. He*λ*ios *α*, Cambridge, UK). Results were expressed as mg of quercetin equivalents/g of extract after interpolating in a calibration curve obtained following the same procedure described above and using quercetin as standard.

### 2.4. CCl_4_-Induced Hepatotoxicity Model in Rats

Male Wistar rats weighing 180–220 g were used in the present study. Experimental protocol followed the guidelines of Norma Oficial Mexicana for the use and care of laboratory animals (NOM-062-ZOO-1999) and for the disposal of biological residues (NOM-087-ECOL-1995). Housing room was maintained under constant conditions of temperature (21 ± 1°C), relative humidity (50–60%), and lighting (12-h light/dark cycle). Filtered air (5 mm particles) was exchanged 18 times/h. Animals were provided with a standard commercial rat chow diet (Harlan Teklad Global diet 2018S sterilized, Harland Teklad, Madison, WI, USA), and reverse osmosis filtered water was used. The animals were divided into seven groups of three rats each one. Group 1 received olive oil (0.1 mL/kg) orally (p.o.) for six days (O.O group). Group 2 received phosphate buffer pH 7.4 (0.1 mL/kg p.o.) for six days (P.B group). Group 3 received 100 mg/kg of acetonic extract p.o, for six days (Ac.E group). Group 4 received 100 mg/kg of of methanolic extract p.o for six days (Me.E group). Groups 1 to 4 were considered as negative control groups. Group 5 was injected with CCl_4_/olive oil (1.5 mL/kg i.p.) the last three days of the experiment. Group 6 received acetonic extract 100 mg/kg p.o for 6 days in combination with CCl_4_/olive oil (1.5 mL/kg i.p.) for the last three days of treatment. Group 7 received methanolic extract 100 mg/kg of p.o for 6 days in combination with CCl_4_/olive oil (1.5 mL/kg i.p.) for the last three days of treatment. Group 8 received quercetin (100 mg/kg body weight) p.o, and Group 9 of rats was exposed to the combination of quercetin 100 mg/kg p.o and CCl_4_ 1.5 mL/kg i.p. for the last three days of treatment. The animals were anesthetized with pentobarbital (0.6 *μ*L/kg) and the blood collected by heart puncture 48 h after the end of the six-day treatment. Tissues (heart, kidney, lungs, and brain) were excised immediately, and a portion was fixed by immersion in buffered formalin and the rest was stored at −70°C for the analysis of antioxidant enzymes. 

### 2.5. Preparation of Tissue Homogenates

Tissues were homogenized in 0.1 M phosphate buffer pH 7.0, with 0.1% Triton X-100, using a Brinkmann Polytron model PT 2000 (Westbury, NY, USA) and centrifuged at 19,000 ×g for 10 min. The supernatant was used for total protein determination [26] and activity of the following antioxidant enzymes: SOD, CAT, GPx, GR, and glutathione transferase (GST) [27].

### 2.6. Biochemical Markers of Tissue Damage in Serum 

Blood samples of each animal were incubated for 45 min at room temperature. Blood serum was separated by centrifugation at 600 ×g for 15 min, and the samples were stored at −20°C. Alkaline phosphatase (ALP), *γ*-Globulin (*γ*-GLOB), serum albumin (ALB), total bilirubin (BB), creatinine (CRE) and creatine kinase (CK) were measured by adaptation of the methodology recommended by the International Federation of Clinical Chemistry (IFCC), with an autoanalyzer (Dimension AR, Dade Behring Inc., Newark, DE, USA).

### 2.7. Estimation of Lipid Peroxidation

Malondialdehyde (MDA) in whole tissue homogenate was measured using a standard curve of trimethoxypropane. The reaction mixture consisted in 0.026 M TBA, 0.211 M HCl, 6.66% trichloroacetic acid, and 1 mM DFO. 200 *μ*L of each tissue homogenate was added to 1,000 *μ*L of reaction mixture, vortexed vigorously and heated at 100°C for 10 min. Mixture was cooled and 1 mL of n-butanol-pyridine (15 : 1) mixture was added. After centrifugation at 1,200 ×g for 10 min. the organic layer was separated and the absorbance was measured at 530 nm. MDA is an end product of lipid peroxidation, which reacts with TBA and the results are expressed in TBARS (nmoles of MDA/mL/mg of protein) [28]. 

### 2.8. Activity of Antioxidant Enzymes 

#### 2.8.1. CAT Assay

CAT activity was assayed at 25°C by a method based on the disappearance of H_2_O_2_ [27]. An aliquot of 5 *μ*L of specific homogenate dilution (1 : 40) was added to 720 *μ*L of 30 mM H_2_O_2_ in 10 mM potassium phosphate solution; the reaction was followed at 240 nm. Under the described conditions, the decomposition of H_2_O_2_ by CAT contained in the samples follows a first-order kinetics as given by the equation *k* = 2.3/*t* log* Ao/A* where *k* is the first-order reaction rate constant, *t* is the time over which the decrease of H_2_O_2_ due to CAT activity was measured (15 s), and* Ao/A* is the optical density at times 0 and 15 s, respectively. The results were expressed in *k*/mg protein.

#### 2.8.2. SOD Assay

SOD activity was assayed by using a previously reported method [27]. A competitive inhibition assay was performed using xanthine-xanthine oxidase system to reduce NBT. The reaction mixture in a final volume of 166 *μ*L contained: 0.122 mM EDTA, 30.6 *μ*M NBT, 0.122 mM xanthine, 0.006% bovine serum albumin and 49 mM sodium carbonate. 33 *μ*L of specific homogenate (1 : 50 dilution) were added to the reaction mixture followed by 30 *μ*L of a xanthine oxidase solution to get a final concentration of 2.5 U/L, and all was incubated at room temperature for 30 min. The reaction was stopped with 66 *μ*L of 0.8 mM cupric chloride and the optical density was read at 560 nm. One hundred percent of NBT reduction was obtained in a tube in which the sample was replaced by distilled water. The amount of protein that inhibited 50% of NBT reduction was defined as one unit of SOD activity. Results were expressed as U/mg protein.

#### 2.8.3. GPx Assay

GPx activity was assayed by a method previously described [27]. The reaction mixture consisted of 50 mM potassium phosphate solution pH 7.0, 1 mM EDTA, 1 mM sodium azide, 0.2 mM NADPH, 25 U/mL of GR, and 1 mM GSH at 25°C. 100 *μ*L of specific homogenate diluted 1 : 10 were added to 800 *μ*L of the reaction mixture and allowed to incubate for 5 min at room temperature before initiation of the reaction by the addition of 32 *μ*L of 2.5 mM H_2_O_2_ solution. Absorbance at 340 nm was recorded for 3 min and the activity was calculated from the slope of these lines as *μ*moles of NADPH oxidized per min taking into account that the millimolar absorption coefficient for NADPH is 6.22. Blank reactions with homogenates replaced by distilled water were subtracted from each assay. One unit of GPx was defined as the amount of enzyme that oxidizes 1 *μ*mol of NADPH/min. The results were expressed as U/mg protein.

#### 2.8.4. GR Assay

GR activity was assayed using GSSG as substrate and measuring the disappearance of NADPH at 340 nm [27]. The reaction mixture consisted of 0.1 M potassium phosphate pH = 7.6, 0.5 mM EDTA, 1.25 mM NADPH, and 0.5 mM GSSG at 25°C. 25 *μ*L of specific dilution of homogenate (1 : 5) were added to 475 *μ*L of reaction mixture. Absorbance at 340 nm was recorded for 3 min and the activity was calculated from the slope of these lines as *μ*moles of NADPH oxidized per min taking into account that the millimolar absorption coefficient for NADPH is 6.22. One unit of GR was defined as the amount of enzyme that oxidizes 1 *μ*mol of NADPH/min. Data were expressed as U/mg protein.

#### 2.8.5. GST Assay

The reaction mixture consisted of 0.05 M phosphate buffer solution pH 6.5, 0.05 M GSH and 0.02 M CDNB. 20 *μ*L of the specific homogenate dilution (1 : 10) were added to 980 *μ*L of the reaction mixture [27]. The changes in the absorbance due to conjugation of the thiol group of GSH to the CDNB substrate were recorded for 3 min at 340 nm and enzyme activity was calculated as *μ*moles of CDNB conjugate formed/min/mg protein using a molar extinction coefficient of 9.6. 

### 2.9. Histopathological Analysis

Tissues were fixed by immersion in buffered formalin (pH 7.4) and embedded in paraffin. For histological analysis, sections (3 *μ*m) were stained with hematoxylin and eosin (H&E) or with periodic acid Schiff's (PAS) to demonstrate polysaccharides, neutral mucopolysaccharide and glycoproteins. The histological profile of the different tissues was taken from 5 randomly selected fields (3 rats per experimental group) recorded using KS-300 software (Carl Zeiss, Jena, Germany). The percentage of damaged areas with histopathological alterations was obtained (magnification 400x). 

### 2.10. Immunohistochemical Analysis of 4-HNE and 3-NT

For immunohistochemistry, tissue sections (3 *μ*m) were deparaffinized and then boiled in Declere (Cell Marque, Hot Springs, AR, USA) to unmask antigen sites; the endogenous activity of peroxidase was quenched with 0.03% H_2_O_2_ in absolute methanol. Tissue sections were incubated overnight at 4°C with 1 : 200 dilution of anti 4-HNE and 1 : 70 dilution of anti 3-NT antibodies in phosphate-buffered saline (PBS). Following removal of the primary antibodies and repetitive rinsing with PBS, slides were incubated with a 1 : 500 dilution of biotinylated goat anti-IgG secondary antibody. Bound antibodies were detected with avidin biotinylated peroxidase complex ABC-kit Vectastain and diaminobenzidine substrate. After appropriate washing in PBS, slides were counterstained with hematoxylin. All sections were incubated under the same conditions with the same concentration of antibodies and in the same running, so the immunostaining was comparable among the different experimental groups. For the negative control, preimmune goat serum was used instead of the primary antibodies. All specimens were examined by light microscopy Axiovert 200 M (Carl Zeiss, Jena, Germany). Five random fields per tissue were studied at a 100x magnification (total area 1,584,000 square microns) comparing the different groups. 

### 2.11. Statistics

Data are expressed as mean ± SD and were analyzed by one-way analysis of variance (ANOVA) followed by a Dunnett's multiple comparison test (GraphPad Prism 4.0 Software, San Diego, CA, USA). A *P* < 0.05 value was considered statistically significant. 

## 3. Results

### 3.1. Phytochemical Study

Acetonic and methanolic extracts of the plant have been previously characterized, and they are known to contain several constituents such as polyacetylenes, catenanes, triterpenes, sterols, sesquiterpenes, flavonoids and flavonoid glycosides [22]. Quercetin was obtained from the methanolic extract and subsequently characterized (Delgado et al., personal communication). Moreover, total phenolic and flavonoid contents, in acetonic and methanolic extracts of *H. inuloides* were estimated based on the method of Folin-Ciocalteu and aluminium chloride using catechin and quercetin as standards, respectively. The total amount of polyphenols contained in acetonic and methanolic extracts were of 19.35 and 50.03 mg/mL of catechin equivalents, respectively. The total flavonoid content was of 0.030 and 0.070 mg/mL of quercetin equivalents in the acetonic and methanolic extracts, respectively. These assays provide a general diagnostic tool of the antioxidant capacity of the extracts.

### 3.2. Effect of Extracts and Quercetin of *H. inuloides* on Biochemical Markers

The results of the effects of extracts and quercetin on CCl_4_-intoxicated rats are shown in Table 1. CCl_4_ treatment significantly increased (*P* < 0.01) the serum levels of ALP, CRE, BB, and CK and decreased the levels of *γ*-GLOB and ALB. The administration of both extracts and quercetin 3 days before and 3 days during CCl_4_ treatment exhibited protection from CCl_4_ toxicity. All of the biological markers of toxicity used indicate that quercetin exhibited a better protective effect followed by methanolic and acetonic extracts in that order, compared with groups of animals that received olive oil and phosphate buffer solution. These results indicate quercetin and the two extracts significantly protected against the increase in ALP, CRE, BB and CK levels as well as the decrease in *γ*-GLOB and ALB levels induced by CCl_4_.

### 3.3. Effect of Extracts and Quercetin of *H. inuloides* on Histopathological Alterations and Immunohistochemical Analysis of 4-HNE and 3-NT

We compared the histoarchitecture of different tissues from control and treated groups of animals using H&E and PAS staining and immunohistochemistry for 3-NT and 4-HNE as markers of damage by oxidative stress and nitrosation, respectively. As shown in Figures 1(a)–1(e), the cardiac muscle fibers revealed no histopathological alterations provoked by any of the treatments used. Fibers are grouped in bundles with connective tissue. Blood capillaries are found in connective tissues and between the cardiac fibers. Each muscle fiber has an acidophilic cytoplasm and a central nucleus in all groups. Negative immunostaining for 3-NT and 4-HNE was observed in heart sections of control group (see Figure 1(a)), in contrast, the animals receiving CCl_4_ were weakly affected (see Figure 1(b)). The experimental groups treated with acetonic and methanolic extracts as well as quercetin, decreased oxidative stress (see Figures 1(c)–1(e)).

 H&E and PAS staining of the kidney (Figures 2(a)–2(e)) revealed, as we expected, entirely normal histological features, glomeruli and tubules have a normal appearance, basement membrane appears orderly in all groups treated. However, a weak staining for 3-NT and 4-HNE was observed in CCl_4_-treated rats (Figure 2(b)) compared to control group (Figure 2(a)). The administration of both extracts and quercetin, in combination with CCl_4_, reversed the weak increase of oxidative stress (see Figures 2(c)–2(e)).

Regarding the analysis of lung tissues: Figure 3 shows representative regions of lung bronchioles, alveoli and arteriole. All animals but those of the CCl_4_ treated group showed normal architecture (see Figures 3(a), and 3(c)–3(e)). The CCl_4_ treated animals showed bronchus associated lymphoid tissue (BALT) significantly more prominent than in other groups (see panel b). The markers of nitrosation and oxidative stress in the animals that received CCl_4_ were weakly affected (see Figure 3(b)) showing elevated immunostaining with respect to control groups (Figure 3(a)). A decrease in the oxidative stress was noted in the experimental groups that received CCl_4_ and acetonic or methanolic extracts and quercetin (see Figures 3(c)-3(d)).

Figures 4(a)–4(e), show representative regions of the brain with normal histological structure. However, we found that compared with the control, the animals that received CCl_4_ were weakly affected in regard to the expression of 3-NT and 4-HNE (see Figure 4(b)). The administration of both extracts and quercetin, in combination with CCl_4_ reversed the elevated expression of markers for nitrosation and oxidative stress (see Figures 4(c)–4(e)). 

### 3.4. Effect of Extracts and Quercetin of *H. inuloides* on Lipid Peroxidation in CCl_4_ Treated Rats

We also verified that CCl_4_ administration increase the TBARS concentrations (expressed as MDA), in the heart 250%, (*P* < 0.01); kidney 170%, (*P* < 0.01); lungs 230%, (*P* < 0.01); and brain 170%, (*P* < 0.05) (Figure 5). The administration of extracts or quercetin reversed the increase of lipid peroxidation caused by CCl_4_ in all tissues. 

### 3.5. Antioxidant Enzymes

In an attempt to obtain more information on the mechanism of protection against CCl_4_ hepatotoxicity by the methanolic extract, we monitored the natural antioxidant cell defenses including the enzymes CAT, SOD, GPx, GR and GST in the different tissues of animals. CCl_4_ administration produced a decrease in the activity of the antioxidant enzymes in every tissue, compared with control groups that received olive oil or phosphate buffer. In the heart tissue (Table 2), GR, CAT and GST activities were reduced by 46–58%, whereas GPx and SOD activities were reduced by 29–36%. 

In kidney tissue SOD and GPx activities were reduced by 41–60%, and GR, GST and CAT had a 21–38% reduced activity (Table 3). 

In lungs (Table 4), CAT, GR and SOD were more affected than in other tissues with a 48–55% reduction followed by GST and GPx with a 35–44% reduction. 

With respect to brain, we analyzed different sections (cerebellum hemispheres and striatum), in order to obtain data regarding the regional specific effects if any (Tables 5, 6 and 7). Our findings showed that the three regions explored showed similar sensibility to the toxic effects of CCl_4_. SOD was the more resistant enzyme with a reduction in its activity of 28–57% in comparison with that obtained for GR, GST; CAT and GPX which showed an activity inhibition of 62–85%. 

## 4. Discussion

ROS contribute to the development of various diseases such as atherosclerosis, diabetes, cancer, neurodegenerative diseases, liver cirrhosis and the ageing process [2, 3, 29]. The use of antioxidant compounds, either natural or synthetic, might help to prevent those conditions and maintain human health. The use of radical scavengers is a good option to cope with those diseases. It is well established that lipid peroxidation is one of the key reactions resulting from the interaction of free radicals and biologic membranes [30, 31].

Since oxidative stress is considered to be the major event responsible for CCl_4_ toxicity, extensive interest has arisen in the investigation of the range of their oxidant power and their harmfulness to different organs. Interest has also arisen in the identification of compounds that are capable of modulating these injuries.* H. inuloides* is a recognized plant with several beneficial health effects that have been used in México for the treatment of postoperative thrombophlebitis and externally for acne, bruises and muscle aches. The major components of acetonic and methanolic extracts of *H. inuloides* have been previously characterized [18, 22]. The methanolic extract is rich in flavonoids and glycoside derivatives, whereas in the acetonic extract, sesquiterpenoids prevail. We previously demonstrated *in vitro *O_2_^●−^ scavenging activity of *H. inuloides *extracts by the EPR method, and we showed that both extracts and the metabolites isolated from *H. inuloides *methanolic extract, scavenged O_2_^●−^, HOCl, H_2_O_2_, ONOO^−^, ^1^O_2_, and OH^●^ very efficiently *in vitro* [18]. *In vivo*, both extracts and quercetin prevented liver oxidative damage induced by CCl_4_ as well as the increase in serum activity of aspartate aminotrasnferase and alanine aminotrasferase [11]. 

In order to obtain more information, we screened the efficacy of the different extracts and quercetin over biochemical markers of tissue damage in serum. The levels of ALP and BB in circulation are sensitive indicators of liver damage; CRE is an indicator of renal failure and CK of the heart damage. Treatment with CCl_4_ caused a significant increase of these markers indicating oxidative injury in the different tissues: *γ*-GLOB and ALB showing decreased levels indicating oxidative injury by CCl_4_. These results are in agreement with increases in ALP, BB, CRE, CK, *γ*-GLOB, and ALB observed by other authors in response to CCl4 [32–35]. The administration of either extract or quercetin 3 days before and 3 days during CCl_4_ treatment prevented the changes in these biomarkers (Table 1).

The lipid solubility of CCl_4_ allows it to cross cell membranes, and when administered it is distributed and deposited to different organs. The time courses of the elimination of CCl_4_ appeared to be governed largely by the rate of blood perfusion and lipid content of the tissue [36]. 

A first level indication of tissue damage induced by CCl_4_ administration was observed in the evaluation of lipid peroxidation. We showed significant increase in MDA levels, a marker of lipid peroxidation in all tissues, 48 h after CCl_4_ treatment. Lipid peroxidation may explain the increased levels of biochemical markers in the blood; the administration of either extracts or quercetin significantly reversed these changes. On the other hand, the basis of CCl4 hepatotoxicity lies in its biotransformation by the cytochrome P450 system giving two free radicals. The first metabolite, CCl_3_^●^, form covalent adducts with lipids and proteins, or it can interact with hydrogen to form chloroform. Aerobically, the trichloromethyl radical can react with oxygen, forming the trichloromethylperoxyl radical CCl_3_OO^●^. Since these enter the circulatory system due to altered permeability of membranes, its rising levels reflected a severe damage to the structural integrity of the tissue [10, 32, 33, 37]. These events lead to membrane lipid peroxidation and the consequent tissue injury [33, 38].

 The administration of the acetonic or methanolic extracts, or quercetin, significantly prevented CCl_4_-induced elevation of MDA indicating the protective activity of *H. inuloides* extracts and quercetin (Figure 5). Interestingly, the exposure of rats to CCl_4_ produced moderate histological changes in the lung, which correlated with the presence of BALT (an ectopic lymphoid tissue that is formed by the presence of an inflammatory response in the lung) [39, 40]; the administration of the acetonic or methanolic extracts or quercetin significantly prevented the formation of BALT (Figure 3). 

On the other hand, CCl_4_-treated groups showed an increase in stress markers 4-HN and 3-NT, in comparison to the untreated groups (Figures 1–4), these processes can affect cognitive function [41]. We hypothesized that the reduced levels of antioxidant enzymes (Tables 2–7) contributed to increased levels of lipoperoxidation, 3NT and 4HN. The administration of either extract or quercetin prevented the adverse effects observed.

It has been reported that SOD, CAT and GST constitute a mutually supportive defense against ROS [1, 2, 6]. In the present work we showed that CCl_4_ induced a significant decrease in the activity of the antioxidant enzymes CAT, SOD, GPx, GR, and GST in the different tissues considered in this study, probably due to protein inactivation by free radicals. Previous studies have demonstrated the different responses of the antioxidant enzymatic systems in different tissues during oxidative stress by CCl_4_ [8, 32, 37, 42–44]. Acetonic and methanolic extracts and quercetin were able to prevent from the decay of antioxidant enzyme activities. This preventive effect could be reflected in the reduction of lipid peroxidation and the improvement of biochemical markers promoted by the extracts and quercetin in all tissues. 

On the other hand, several studies have shown that natural antioxidant defense system has limited capacity in the brain as compared to peripheral tissues. Such is the case with glutathione (GSH), the major intracellular antioxidant present ubiquitously in the mM range throughout the brain. GSH detoxifies intracellular H_2_O_2_ to H_2_O and O_2_ via subsequent oxidation to glutathione disulfide (GSSG) by the enzyme glutathione peroxidase (GPx). GSSG is recycled to GSH via glutathione reductase (GR) [45]. It has been reported that the brain contains small amounts of CAT activity, and different brain regions contain different activities of antioxidant enzymes [46], including GPx and SOD [47]. Our results agree in part with this notion since the different parts of cerebral tissues evaluated showed ten times less CAT activity than kidney and lung and 100 times less activity than heart. Additionally, GR activity in cerebral tissues is one order of magnitude lower than that observed in heart, kidney and lung (Tables 2–7). No big differences were noted in enzyme activity between the three cerebral regions studied.

Manoli et al. [48] and Baek et al. [49] concluded that the vulnerability to oxidative stress in the brain is region-specific and is dependent on local endogenous iron-catalyzed Fenton reaction or by the Haber-Weiss reaction. Other authors reported that regions like cortex, hypothalamus, hippocampus, and striatum are more susceptible to oxidative damage in comparison with cerebellum. In this study, histological analysis showed more damage in cerebellum, followed by striatum and hemispheres, this damage was reversed by quercetin and both extracts [50, 51].

Lipoperoxidation has been shown to be involved in excitotoxicity of neurons [52, 53], leading to the increase of iron levels and generating peroxyl/alkoxyl radicals potentiating lipid peroxidation by a positive feedback [54]. Since the treatment with either extract or quercetin normalized the activity of CAT, SOD, GPx, and GR in different regions of the brain, it would prevent lipoperoxidation and the subsequent adverse effects.

The beneficial effects of *H. inuloides* extracts and quercetin against CCl_4_ toxicity on the several tissues considered in this study could be due in part to its hepatoprotection reported previously [11]. Liver is the main target of CCl_4_ toxicity, and its elevated activity in CYP2E1 leads to the production of toxic free radicals. Nevertheless, hepatic Phase II enzymes and glutathione participate in CCl_4_ metabolite detoxification. In this way, free radicals could be inactivated by *H. inuloides* components living a functional liver to continue its detoxification role. On the other hand, CYP2E1 is present in the tissues considered in this work; therefore, in situ metabolism of CCl_4_ could take place leading to the production of the toxic metabolites and the modulation of the antioxidant enzymes. It remains to determine the role of each organ detoxifying mechanisms versus overall liver detoxification achieved.

## 5. Conclusions

These results indicate that either extracts or quercetin could protect against lipid peroxidation, maintaining the basal antioxidant activity and the levels of different biochemical parameters; this effect is attributed to its free radical scavenger properties. We suggest that methanolic and acetonic extracts and quercetin of *H. inuloides* could confer protection against acute tissue injury induced by CCl_4_ and other environmental contaminants or biological agents capable of inducing free radicals. Results reported here support the attributed biomedical properties of this plant.

## Figures and Tables

**Figure 1:** Histopathological and immunohistochemical analysis in cardiac muscle sections (3 *μ*m) obtained 48 h after last day of treatment (*n* = 3): (a) control rats, (b) CCl_4_-treated rats, (c) CCl_4_-treated rats with Ac.E, (d) CCl_4_-treated rats with Me.E, and (e) CCl_4_-treated rats with quercetin, magnification 100x.

**Figure 2:** Histopathological and immunohistochemical analysis in kidney tissue sections (3 *μ*m) obtained 48 h after last day of treatment (*n* = 3): (a) control rats, (b) CCl_4_-treated rats, (c) CCl_4_-treated rats with Ac.E, (d) CCl_4_-treated rats with Me.E, and (e) CCl_4_-treated rats with quercetin, magnification 100x.

**Figure 3:** Histopathological and immunohistochemical analysis in lung tissue sections (3 *μ*m) obtained 48 h after last day of treatment (*n* = 3): (a) control rats, (b) CCl_4_-treated rats, (c) CCl_4_-treated rats with Ac.E, (d) CCl_4_-treated rats with Me.E, and (e) CCl_4_-treated rats with quercetin, magnification 100x. The arrows show the formation of BALTS.

**Figure 4:** Histopathological and immunohistochemical analysis in brain tissue sections (3 *μ*m) obtained 48 h after last day of treatment (*n* = 3): (a) control rats, (b) CCl_4_-treated rats, (c) CCl_4_-treated rats with Ac.E, (d) CCl_4_-treated rats with Me.E, (e) CCl_4_-treated rats with quercetin, magnification 100x.

**Figure 5:** Effect of acetonic and methanolic extracts of *H inuloides* and quercetin on increased MDA levels induced by CCl_4_: (a) heart, (b) kidney, (c) lungs, and (d) brain. O.O, olive oil; P.B, phosphate buffer; Ac. E, acetonic extract; Me. E, methanolic extract; Quer, quercetin; CCl_4_, carbon tetrachloride. Rats were sacrificed 48 h after the end of treatment. MDA determination was performed three times, in triplicate, and the values represent the mean ±S.D of 9 determinations. *P < 0.01 versus O.O, P.B, Ac.E, Me.E, Quer, CCl_4_ + Me.E and CCl_4_ + Ac. E, ^#^ *P* < 0.05 versus CCl_4_.

**Table 1:** Effect of extracts of *H. inuloides* and quercetin, on serum clinical chemistry parameters of Wistar rats untreated and CCl_4_ treated at dose of 1.5 mL/kg for three consecutive days.

Group	ALP	*γ*-GLOB	ALB	BB	CRE	CK
O.O	216.6 ± 7	7.0 ± 1.0	1.18 ± 0.15	1.30 ± 0.20	0.40 ± 0.02	100.00 ± 13
P.B	215.3 ± 12	6.0 ± 1.3	1.10 ± 0.05	1.40 ± 0.10	0.42 ± 0.03	110.54 ± 15
Ac.E	183.0 ± 8	4.8 ± 0.59	1.16 ± 0.15	1.90 ± 0.20	0.49 ± 0.04	171.05 ± 12
Me.E	204.3 ± 31	5.25 ± 1.0	1.03 ± 0.05	1.70 ± 0.10	0.47 ± 0.02	157.47 ± 10
Quer	159.0 ± 14	4.49 ± 0.54	1.05 ± 0.07	1.60 ± 0.10	0.45 ± 0.03	105.62 ± 9
CCl_4_	271.6 ± 7^*α*,+^	1.5 ± 0.30*	0.65 ± 0.05*	3.8 ± 0.10*	0.90 ± 0.04*	321.25 ± 15*
Ac.E + CCl_4_	234.0 ± 6	5.50 ± 0.57	0.96 ± 0.05	2.0 ± 0.10	0.47 ± 0.03	212.48 ± 15
Me.E + CCl_4_	227.3 ± 5	5.66 ± 0.47	0.99 ± 0.02	1.50 ± 0.10	0.45 ± 0.01	197.87 ± 13
Quer + CCl_4_	121.5 ± 22	5.2 ± 0.15	1.05 ± 0.07	1.10 ± 0.10	0.44 ± 0.02	149.73 ± 19

Alkaline phosphatase (ALP) (U/L), *γ*-globulin (*γ*-GLOB) (g/dL), serum albumin (ALB) (g/dL), total bilirubin (BB) (*μ*mol/L), creatinine (CRE) (*μ*mol/L), creatine kinase (CK) (U/L). *P < 0.01 versus all groups; ^*α*^ *P* < 0.01 versus O.O, P.B, Ac.E, Me.E, Quer, Ac.E + CCl_4_, Quer + CCl_4_; ^+^ *P* < 0.05 versus Me.E + CCl_4_. Each determination was performed twice, in triplicate, and the values represent the mean ± SD. *n* = 3.

**Table 2:** Effect of extracts of *H. inuloides*, and quercetin on the antioxidant enzymes in heart tissue of Wistar rats untreated and CCl_4_ treated at dose of 1.5 mL/kg for three consecutive days.

Group	CAT k/mg protein	SOD U/mg protein	GPx U/mg protein	GR U/mg protein	GST *μ*mol CDNB/min/mg protein
O.O	1.66 ± 0.05	55.28 ± 2	0.036 ± 0.001	0.179 ± 0.03	0.552 ± 0.02
P.B	1.57 ± 0.01	40.32 ± 1	0.041 ± 0.005	0.174 ± 0.04	0.324 ± 0.03
Ac.E	1.31 ± 0.01	35.26 ± 3	0.033 ± 0.002	0.161 ± 0.01	0.315 ± 0.02
Me.E	1.38 ± 0.01	41.95 ± 2	0.047 ± 0.001	0.163 ± 0.03	0.513 ± 0.02
Quer	1.55 ± 0.02	38.22 ± 2	0.051 ± 0.001	0.161 ± 0.10	0.368 ± 0.02
CCl_4_	1.11 ± 0.01*	23.29 ± 3*	0.027 ± 0.001*	0.095 ± 0.01*	0.109 ± 0.03^●, #^
CCl_4_ + Ac.E	1.33 ± 0.02	31.20 ± 1	0.031 ± 0.002	0.155 ± 0.06	0.369 ± 0.03
CCl_4_ + Me.E	1.35 ± 0.03	33.97 ± 2	0.036 ± 0.001	0.163 ± 0.07	0.569 ± 0.03
CCl_4_ + Quer	1.38 ± 0.04	35.14 ± 3	0.048 ± 0.001	0.156 ± 0.01	0.516 ± 0.03

Olive oil (O.O), 0.1 mL/kg; phosphate buffer (P.B), 0.1 mL/kg; acetonic extract (Ac.E) 100 mg/kg p.o; methanolic extract (Me.E) 100 mg/kg p.o; quercetin (Quer)/P.B, (100 mg/kg/200 *μ*L p.o); Ac.E + CCl_4_, corresponded to acetonic extract for 6 days in combination with CCl_4_ (100 mg/kg p.o, 1.5 mL/kg i.p); Me.E + CCl_4_, corresponded to methanol extract for 6 days in combination with CCl_4 _(100 mg/kg p.o, 1.5 mL/kg i.p); Quer + CCl_4_, (100 mg/kg/200 *μ*L p.o, 1.5 mL/kg i.p) corresponded to quercetin for 6 days in combination with CCl_4_ for the last three days of treatment. *P < 0.01 versus all groups, ^●^ *P* < 0.05 versus P.B, and ^#^ *P* < 0.01 versus O.O, P.B. Ac.E, Me.E, Quer, CCl_4_ + Me.E, CCl_4 _+ Ac.E, CCl_4 _+ Quer. Each determination was performed twice, in triplicate, and the values represent the mean ± SD. *n* = 3.

**Table 3:** Effect of extracts of *H. inuloides* and quercetin on the antioxidant enzymes in kidney tissue of Wistar rats untreated and CCl_4_-treated at dose of 1.5 mL/kg for three consecutive days.

Group	CAT k/mg protein	SOD U/mg protein	GPx U/mg protein	GR U/mg protein	GST *μ*mol conjugate CDNB/min/mg protein
O.O	0.156 ± 0.01	71.35 ± 2	0.046 ± 0.01	0.125 ± 0.01	0.331 ± 0.01
P.B	0.136 ± 0.02	74.76 ± 2	0.042 ± 0.01	0.112 ± 0.01	0.309 ± 0.01
Ac.E	0.128 ± 0.01	64.61 ± 3	0.037 ± 0.02	0.129 ± 0.01	0.321 ± 0.01
Me.E	0.144 ± 0.02	69.84 ± 1	0.043 ± 0.01	0.152 ± 0.01	0.354 ± 0.03
Quer	0.146 ± 0.01	70.70 ± 2	0.038 ± 0.02	0.147 ± 0.02	0.340 ± 0.01
CCl_4_	0.091 ± 0.01^●,+^	42.70 ± 2*	0.018 ± 0.01*	0.088 ± 0.009^#,†^	0.254 ± 0.03*
CCl_4 _+ Ac.E	0.135 ± 0.03	54.30 ± 2	0.035 ± 0.02	0.118 ± 0.01	0.325 ± 0.01
CCl_4 _+ Me.E	0.138 ± 0.02	57.17 ± 1	0.041 ± 0.01	0.129 ± 0.01	0.329 ± 0.03
CCl_4 _+ Quer	0.150 ± 0.01	68.84 ± 2	0.034 ± 0.02	0.140 ± 0.01	0.339 ± 0.01

Olive oil (O.O), 0.1 mL/kg; phosphate buffer (P.B), 0.1 mL/kg; acetonic extract (Ac.E) 100 mg/kg p.o; methanolic extract (Me.E) 100 mg/kg p.o; quercetin (Quer)/P.B, (100 mg/kg/200 *μ*L p.o); Ac.E + CCl_4_, corresponded to acetonic extract for 6 days in combination with CCl_4_ (100 mg/kg p.o, 1.5 mL/kg i.p); Me.E + CCl_4_, corresponded to methanol extract for 6 days in combination with CCl_4 _ (100 mg/kg p.o, 1.5 mL/kg i.p); Quer + CCl_4_, (100 mg/kg/ 200 *μ*L p.o, 1.5 mL/kg i.p) corresponded to quercetin for 6 days in combination with CCl_4_ for the last three days of treatment. ^●^ *P* < 0.01 versus O.O, P.B, Me.E, Que, CCl_4_ + Ac.E, CCl_4_ + Me.E, CCl_4_ + Quer, ^+^ *P* < 0.05 versus, Ac.E, *P < 0.01 versus. all groups, ^ #^ *P* < 0.01 versus O.O, Ac.E, Me.E, Que, CCl_4_ + Ac.E, CCl_4_ + Me.E, CCl_4_ + Quer., ^†^ *P* < 0.05 versus P.B. Each determination was performed twice, in triplicate, and the values represent the mean ± SD. *n* = 3.

**Table 4:** Effect of extracts of *H. inuloides* and quercetin, on the antioxidant enzymes in lung tissue of Wistar rats untreated and CCl_4_ treated at dose of 1.5 mL/kg for three consecutive days.

Group	CAT k/mg protein	SOD U/mg protein	GPx U/mg protein	GR U/mg protein	GST *μ*mol conjugado CDNB/min/mg protein
O.O	0.120 ± 0.01	51.15 ± 1.3	0.036 ± 0.001	0.105 ± 0.012	0.241 ± 0.002
P.B	0.100 ± 0.02	48.36 ± 1.5	0.032 ± 0.001	0.101 ± 0.014	0.229 ± 0.003
Ac.E	0.090 ± 0.01	44.31 ± 1.1	0.027 ± 0.001	0.090 ± 0.011	0.211 ± 0.002
Me.E	0.095 ± 0.01	49.14 ± 0.9	0.023 ± 0.002	0.095 ± 0.010	0.214 ± 0.003
Quer	0.101 ± 0.01	45.10 ± 1.1	0.030 ± 0.001	0.100 ± 0.014	0.226 ± 0.001
CCl_4_	0.056 ± 0.01^●,+^	22.70 ± 1.2*	0.019 ± 0.001*	0.053 ± 0.011^#,‡^	0.152 ± 0.004*
CCl_4 _+ Ac.E	0.080 ± 0.001	34.40 ± 1.7	0.025 ± 0.002	0.082 ± 0.014	0.198 ± 0.003
CCl_4 _+ Me.E	0.089 ± 0.01	37.17 ± 1.2	0.024 ± 0.001	0.088 ± 0.007	0.209 ± 0.003
CCl_4 _+ Quer	0.092 ± 0.01	40.84 ± 2.0	0.022 ± 0.001	0.092 ± 0.005	0.229 ± 0.001

Olive oil (O.O), 0.1 mL/kg; phosphate buffer (P.B), 0.1 mL/kg; acetonic extract (Ac.E) 100 mg/kg p.o; methanolic extract (Me.E) 100 mg/kg p.o; quercetin (Quer)/P.B, (100 mg/kg/200 *μ*L p.o); Ac.E + CCl_4_, corresponded to acetonic extract for 6 days in combination with CCl_4_ (100 mg/kg p.o, 1.5 mL/kg i.p); Me.E + CCl_4_, corresponded to methanol extract for 6 days in combination with CCl_4_ (100 mg/kg p.o, 1.5 mL/kg i.p); Quer + CCl_4_, (100 mg/kg/200 *μ*L p.o, 1.5 mL/kg i.p) corresponded to quercetin for 6 days in combination with CCl_4_ for the last three days of treatment. ^●^ *P* < 0.01 versus O.O, P.B. Ac.E, Me.E, Quer, CCl_4_ + Me.E, Ac.E, CCl_4_ + Quer,^ +^ *P* < 0.05 versus CCl_4_ + Ac.E, *P < 0.01 versus all groups, ^#^ *P* < 0.01 versus O.O, P.B. Ac.E, Me.E, Quer, CCl_4_ + Me.E, CCl_4_ + Quer, ^‡^ *P* < 0.05 versus CCl_4_ + Ac.E. Each determination was performed twice, in triplicate and the values represent the mean ± SD. *n* = 3.

**Table 5:** Effect of extracts of *H. inuloides* and quercetin, on the antioxidant enzymes in cerebellum tissue of Wistar rats untreated and CCl_4_ treated at dose of 1.5 mL/kg for three consecutive days.

Group	CAT k/mg protein	SOD U/mg protein	GPx U/mg protein	GR U/mg protein	GST *μ*mol CDNB/min/mg protein
O.O	0.074 ± 0.005	76.31 ± 4.0	0.040 ± 0.001	0.032 ± 0.001	0.187 ± 0.002
P.B	0.064 ± 0.001	57.07 ± 1.4	0.038 ± 0.002	0.022 ± 0.002	0.160 ± 0.003
Ac.E	0.051 ± 0.005	50.33 ± 1.7	0.030 ± 0.001	0.016 ± 0.03	0.152 ± 0.002
Me.E	0.057 ± 0.003	55.75 ± 1.4	0.034 ± 0.001	0.017 ± 0.001	0.154 ± 0.004
Quer	0.059 ± 0.003	55.10 ± 1.1	0.036 ± 0.001	0.019 ± 0.004	0.146 ± 0.004
CCl_4_	0.028 ± 0.002*	40.88 ± 1.8*	0.015 ± 0.001*	0.009 ± 0.003*	0.112 ± 0.005*
CCl_4 _+ Ac.E	0.047 ± 0.002	34.40 ± 1.7	0.035 ± 0.002	0.011 ± 0.003	0.135 ± 0.004
CCl_4 _+ Me.E	0.053 ± 0.003	37.17 ± 1.3	0.037 ± 0.001	0.017 ± 0.001	0.140 ± 0.005
CCl_4 _+ Quer	0.060 ± 0.003	50.98 ± 1.4	0.033 ± 0.002	0.018 ± 0.003	0.143 ± 0.007

Olive oil (O.O), 0.1 mL/kg; phosphate buffer (P.B), 0.1 mL/kg; acetonic extract (Ac.E) 100 mg/kg p.o; methanolic extract (Me.E) 100 mg/kg p.o; quercetin (Quer)/P.B, (100 mg/kg/200 *μ*L p.o); Ac.E + CCl_4_, corresponded to acetonic extract for 6 days in combination with CCl_4_ (100 mg/kg p.o, 1.5 mL/kg i.p); Me.E + CCl_4_, corresponded to methanol extract for 6 days in combination with CCl_4 _(100 mg/kg p.o, 1.5 mL/kg i.p); Quer + CCl_4_, (100 mg/kg/200 *μ*L p.o, 1.5 mL/kg i.p) corresponded to quercetin for 6 days in combination with CCl_4_ for the last three days of treatment.*P < 0.01 versus all groups. Each determination was performed twice, in triplicate, and the values represent the mean ± SD. *n* = 3.

**Table 6:** Effect of extracts of *H. inuloides* and quercetin, on the antioxidant enzymes in hemispheres tissue of Wistar rats untreated and CCl_4_ treated at dose of 1.5 mL/kg for three consecutive days.

Group	CAT k/mg protein	SOD U/mg protein	GPx U/mg protein	GR U/mg protein	GST *μ*molCDNB/min/mg protein
O.O	0.013 ± 0.001	67.13 ± 4.0	0.046 ± 0.006	0.023 ± 0.003	0.178 ± 0.002
P.B	0.012 ± 0.005	86.41 ± 0.50	0.045 ± 0.008	0.021 ± 0.002	0.150 ± 0.003
Ac.E	0.010 ± 0.003	85.24 ± 1.2	0.040 ± 0.002	0.016 ± 0.004	0.132 ± 0.009
Me.E	0.011 ± 0.002	80.83 ± 1.4	0.041 ± 0.003	0.018 ± 0.003	0.146 ± 0.005
Quer	0.011 ± 0.001	80.96 ± 1.1	0.043 ± 0.003	0.021 ± 0.003	0.151 ± 0.006
CCl_4_	0.003 ± 0.002^+^	48.04 ± 1.8*	0.011 ± 0.001*	0.008 ± 0.002^●,‡^	0.065 ± 0.008^+^
CCl_4 _+ Ac.E	0.006 ± 0.002	75.64 ± 0.04	0.039 ± 0.001	0.015 ± 0.003	0.135 ± 0.004
CCl_4 _+ Me.E	0.010 ± 0.002	82.31 ± 1.74	0.040 ± 0.001	0.018 ± 0.002	0.140 ± 0.005
CCl_4 _+ Quer	0.010 ± 0.003	82.85 ± 1.61	0.042 ± 0.001	0.019 ± 0.002	0.143 ± 0.007

Olive oil (O.O), 0.1 mL/kg; phosphate buffer (P.B), 0.1 mL/kg; acetonic extract (Ac.E) 100 mg/kg p.o; methanolic extract (Me.E) 100 mg/kg p.o; quercetin (Quer)/P.B, (100 mg/kg/200 *μ*L p.o); Ac.E + CCl_4_, corresponded to acetonic extract for 6 days in combination with CCl_4_ (100 mg/kg p.o, 1.5 mL/kg i.p); Me.E + CCl_4_, corresponded to methanol extract for 6 days in combination with CCl_4_ (100 mg/kg p.o, 1.5 mL/kg i.p); Quer + CCl_4_, (100 mg/kg/200 *μ*L p.o, 1.5 mL/kg i.p) corresponded to quercetin for 6 days in combination with CCl_4_ for the last three days of treatment. ^+^ *P* < 0.05 versus all groups, *P < 0.01 versus all groups, ^●^ *P* < 0.01 versus O.O, P.B. Ac.E, Me.E, Quer, CCl_4_ + Me.E, CCl_4_ + Quer, ^‡^ *P* < 0.05 versus CCl_4_ + Ac.E. Each determination was performed twice, in triplicate, and the values represent the mean ± SD. *n* = 3.

**Table 7:** Effect of extracts of *H. inuloides* and quercetin, on the antioxidant enzymes in striatum tissue of Wistar rats untreated and CCl_4_ treated at dose of 1.5 mL/kg for three consecutive days.

GROUP	CAT k/mg protein	SOD U/mg protein	GPx U/mg protein	GR U/mg protein	GST *μ*mol CDNB/min/mg protein
O.O	0.017 ± 0.004	67.13 ± 4.0	0.055 ± 0.006	0.033 ± 0.003	0.175 ± 0.003
P.B	0.014 ± 0.003	57.07 ± 1.4	0.053 ± 0.003	0.030 ± 0.008	0.167 ± 0.005
Ac.E	0.011 ± 0.002	50.33 ± 1.7	0.049 ± 0.007	0.027 ± 0.003	0.157 ± 0.009
Me.E	0.013 ± 0.002	55.75 ± 1.4	0.051 ± 0.001	0.030 ± 0.002	0.165 ± 0.007
Quer	0.014 ± 0.003	55.10 ± 1.1	0.055 ± 0.004	0.033 ± 0.006	0.166 ± 0.002
CCl_4_	0.004 ± 0.001*	28.88 ± 1.8*	0.018 ± 0.002*	0.005 ± 0.002*	0.035 ± 0.009*
CCl_4 _+ Ac.E	0.010 ± 0.003	35.40 ± 1.2	0.043 ± 0.004	0.023 ± 0.004	0.155 ± 0.005
CCl_4 _+ Me.E	0.012 ± 0.005	37.17 ± 1.3	0.048 ± 0.005	0.027 ± 0.005	0.161 ± 0.003
CCl_4 _+ Quer	0.013 ± 0.004	50.98 ± 1.4	0.052 ± 0.007	0.031 ± 0.005	0.163 ± 0.002

Olive oil (O.O), 0.1 mL/kg; phosphate buffer (P.B), 0.1 mL/kg; acetonic extract (Ac.E) 100 mg/kg p.o; methanolic extract (Me.E) 100 mg/kg p.o; quercetin (Quer)/P.B, (100 mg/kg/200 *μ*L p.o); Ac.E + CCl_4_, corresponded to acetonic extract for 6 days in combination with CCl_4_ (100 mg/kg p.o, 1.5 mL/kg i.p); Me.E + CCl_4_, corresponded to methanol extract for 6 days in combination with CCl_4_ (100 mg/kg p.o, 1.5 mL/kg i.p); Quer + CCl_4_, (100 mg/kg/200 *μ*L p.o, 1.5 mL/kg i.p) corresponded to quercetin for 6 days in combination with CCl_4_ for the last three days of treatment. *P < 0.01 versus all groups. Each determination was performed twice, in triplicate, and the values represent the mean ± SD. *n* = 3.
